# Expression and Regulation Network of HDAC3 in Acute Myeloid Leukemia and the Implication for Targeted Therapy Based on Multidataset Data Mining

**DOI:** 10.1155/2022/4703524

**Published:** 2022-03-14

**Authors:** Minhua Li, Feifei Lan, Chen Li, Ning Li, Xiaojie Chen, Yueyuan Zhong, Yue Yang, Yingqi Shao, Yi Kong, Xinming Li, Danny Wu, Jingyu Zhang, Wenqing Chen, Zesong Li, Xiao Zhu

**Affiliations:** ^1^School of Laboratory Medicine, Hangzhou Medical College, Hangzhou, China; ^2^Zhu's Group, Guangdong Medical University, Zhanjiang, China; ^3^Medical Genetics Center, Guangdong Women and Children Hospital, Guangzhou, China; ^4^Department of Biology, Chemistry, Pharmacy, Free University of Berlin, 14195 Berlin, Germany; ^5^The First Affiliated Hospital of Shenzhen University, Shenzhen Second People's Hospital (Shenzhen Institute of Translational Medicine), Shenzhen, China

## Abstract

**Background:**

Histone deacetylase 3 (HDAC3) plays an important role in the development and progression of a variety of cancers, but its regulatory mechanism in acute myeloid leukemia (LAML) is not entirely understood.

**Methods:**

We analyzed the expression of HDAC3 in normal and cancerous tissues using Oncomine, UALCAN, and GEO databases. Changes of the HDAC3 gene were analyzed by cBioPortal. The genes coexpressed with HDAC3 were analyzed by WebGestalt, and the predicted signaling pathways in KEGG were discussed.

**Results:**

We discovered that the expression of HDAC3 was elevated in some types of acute myeloid leukemia. The HDAC3 gene has a strong positive correlation with SLC25A5, NDUFA2, Cox4I1, and EIF3K, which regulate cell growth and development. HDAC3 transcription is higher in patients with FLT3 mutation than in healthy people. HDAC3 can be directly involved in regulating the thyroid hormone signaling pathway. MEF2D is directly involved in the cGMP-PKG signaling pathway, and the HDAC3 gene has a strong synergistic relationship with MEF2D. HDAC3 is indirectly involved in the cGMP-PKG signaling pathway, thereby indirectly regulating the expression levels of p53 and p21 genes in patients with LAML. Genomics of Drug Sensitivity in Cancer (GDSC) database analysis revealed that the application of the HDAC3 inhibitor can inhibit the proliferation of leukemia cells.

**Conclusions:**

Therefore, our data suggest that HDAC3 may be a possible therapeutic target for acute myeloid leukemia.

## 1. Introduction

Acute myeloid leukemia (LAML) is a group of highly heterogeneous hematologic tumors caused by malignant clonal proliferation, dysdifferentiation, and blocked apoptosis of hematopoietic stem cells [1]. Epidemiological surveys show that acute myeloid leukemia is the most common type of adult leukemia and about 25% of adult leukemia patients worldwide belong to LAML and the incidence increases with age [2]. There has been a great deal of research into acute myeloid leukemia over the past few decades, but little progress has been made. The current treatment for LAML is mainly chemotherapy with anthracycline plus cytiside arabinoside [3]. Anticancer drugs used in chemotherapy can largely kill abnormal leukemia cells in the blood and bone marrow, but at the same time, they also kill part of the normal cells that grow rapidly, so patients have a low long-term survival rate and poor therapeutic efficacy and recovery [4]. The 2-year survival rate was approximately 35% for most patients, and the 2-year survival rate of some subtypes is even below 5% [5]. Acute myeloid leukemia has a long treatment cycle, painful treatment process, high recurrence rate, and low survival rate, which bring great pain and economic burden to patients and their families [6]. Therefore, according to the heterogeneity of LAML patients, screening effective drug targets for the treatment of acute myeloid leukemia provides a new possibility.

Histone deacetylase (HDAC) is a kind of regulation of histone acetylation by protease, the enzyme can be removed from lysine acetyl, and most of the work, by protein complexes formed, is the modification of the chromosome structure and gene expression regulation and control important regulatory factors [7, 8]. Conversely, deacetylation can also lead to transcriptional inhibition and impaired hematopoietic differentiation. HDAC is involved in a variety of physiological and pathological processes such as cell survival, proliferation, angiogenesis, inflammation, and immunity and is also involved in multiple cell biological signal transduction pathways, which also play an important role in the occurrence and development of malignant tumors. Histone deacetylase 3 (HDAC3) is a form of HDAC. HDAC3 in the use of other types of HDAC homology search was found for the first time [9], and then, the abnormal expression in multiple myeloma, liver cancer, and other malignant tumors was confirmed [10–12].

HDAC3 can promote the occurrence and development of leukemia by activating *β*-catenin, protein kinase B (AKT), and other cytokines. The regulatory effect of histone deacetylase inhibitors (HDACi) on leukemia-related transcription factor *β*-catenin, Wilms tumor (WT1), and myeloma oncogene (MYC) was detected by Western blotting. The results showed that the expression and activity of these cytokines were related to the occurrence of the disease, poor karyotype, and poor prognosis. The application of HDCA3 inhibitors can inhibit the growth of cancer cells and disrupt the expression of tumor-related proteins [13].

These results suggest that HDAC3 may be a new drug target. Therefore, we used multidimensional analysis to study HDAC3 changes in LAML and related gene function networks, aiming to provide a new diagnostic and therapeutic strategy for acute myeloid leukemia.

## 2. Methods

### 2.1. Oncomine Database Analysis

Oncomine (http://www.oncomine.org) is currently the world's largest oncogene chip database and integrated data mining platform. It combines The Cancer Genome Atlas (TCGA), Gene Expression Omnibus (GEO), ArrayExpress, and other databases and is assembled after a series of processing, standardization, and analysis [14]. To date, nearly 800 gene expression databases and more than 90,000 cancer and normal tissue samples have been collected [15]. In this study, we drew on a series of studies on acute myeloid leukemia, including Andersson leukemia, Valk leukemia, Stegmaier leukemia, Haferlach leukemia, and TCGA leukemia 2. We compared the expression of HDAC3 in normal tissue cells with that in acute myeloid leukemia and then analyzed the difference in HDAC3 expression; *p* < 0.05 was statistically significant.

### 2.2. UALCAN Database Analysis

UALCAN is an effective cancer data online analysis, and the mining site is mainly based on the TCGA-related cancer data in the database; the database can be used according to different types of cancer, cancer classification, gender, and race to query the clinical pathological characteristics of gene expression in cancer and normal tissue sample analysis [16]. We used it to further determine the expression level of HDAC3 in LAML in TCGA samples and the difference of the gene expression level in patients with different survival years and then analyze the impact of HDAC3 expression difference on patient survival. UALCAN is publicly available at http://ualcan.path.uab.edu.

### 2.3. cBioPortal Database Analysis

cBioPortal (http://www.cbioportal.org) is a comprehensive open network platform based on TCGA database, which integrates data mining, data integration, and visualization and currently covers 290 cancer studies [17, 18]. We used cBioPortal to analyze HDAC3 and its related genes, and the label oncoPrint showed an overview of the genetic changes of HDAC3 in each sample, and the label mutual exclusivity showed the pair interaction relationship between HDAC3 and its related genes.

### 2.4. STRING Analysis

STRING database (http://string-db.org/) is an online search database for known protein-protein interactions (PPI) [19]. We performed PPI network analysis on HDAC3 and its related genes to explore their direct or indirect interactions.

### 2.5. LinkedOmics Database Analysis

LinkedOmics is a multiomics database containing 32 TCGA cancer types [20]. It includes three analysis modules: LinkFinder, LinkInterpreter, and LinkCompare. We used the LinkFinder module to study the differential expression of HDAC3-related genes in the TCGA LAML cohort, and the results were statistically analyzed by Pearson's correlation coefficient. All results are shown in volcanic, heat, or scatter maps. LinkedOmics is freely available at http://www.linkedomics.org.

### 2.6. WebGestalt Database Analysis

WebGestalt is a feature-rich tool for gene analysis. WebGestalt supports 12 organisms, 342 gene identifiers, and 155 functional categories [21]. Functional enrichment analysis of genes plays an important role in the biological interpretation of high-throughput omics data [22]. We performed Gene Ontology (GO) and Kyoto Encyclopedia of Genes and Genomes (KEGG) pathway enrichment analysis on 25 genes related to HDAC3 and searched for possible biological functions of HDAC3 through bioinformatics methods combined with big data from the database. GO annotation is divided into three parts: the cellular component (CC), biological process (BP), and molecular function (MF).

### 2.7. Genomics of Drug Sensitivity in Cancer (GDSC) Database Analysis

Genomics of Drug Sensitivity in Cancer database (http://www.cancerRxgene.org) is the world's largest public database for obtaining information on drug sensitivity and molecular markers of drug responses in cancer cells [23]. We used the GDSC database to find the HDAC3-targeted drug entinostat and predicted the resistance of entinostat to tumors with high HDAC3 expression.

## 3. Results

### 3.1. Expression of HDAC3 in Acute Myeloid Leukemia

We first analyzed the deoxyribonucleic acid (DNA) copy number variation (CNV) and messenger RNA (mRNA) transcription levels of HDAC3 in acute myeloid leukemia using Oncomine database to investigate the expression of HDAC3 in acute myeloid leukemia. In the Andersson leukemia dataset, HDAC3 over expression was found in LAML compared with normal bone marrow with a fold change of 1.729 in acute myeloid leukemia (*p* < 0.05). However, compared with normal tissue cells, DNA copy number variations of HDAC3 and mRNA expression levels in Valk, Stegmaier, and Haferlach leukemia datasets were not significantly different in acute myeloid leukemia (*p* > 0.05) (Figure 1). The UALCAN database was used to further analyze the differential expression of HDAC3 in acute myeloid leukemia. The results showed that the expression level of HDAC3 was different in different subtypes of acute myeloid leukemia. The expression level of HDAC3 was relatively high in the M5 subtype and relatively low in the M7 subtype (Figure 2(a)). The HDAC3 transcription level in patients with FMS-like tyrosine kinase 3 (FLT3) gene mutation was higher than that in healthy people, *p* = 5.521800*E* − 02 (Figure 2(e)). From survival analysis of LAML patients, patients with high HDAC3 mRNA expression levels had a shorter survival time, while patients with medium-/low-HDAC3 mRNA expression levels had a longer survival time (*p* < 0.05). HDAC3 mRNA transcription levels were higher in various types of malignant tumors than in normal tissues (Figure 3). Taken together, HDAC3 may be a potential therapeutic target for acute myeloid leukemia.

We used cBioPortal to analyze HDAC3 alterations in the TCGA LAML samples and found that 24 of 1008 (2.4%) samples had HDAC3 mutations (Figure S1-A). We next wanted to determine the biological interaction network of HDAC3 in LAML. UALCAN is used to find a gene set related to HDAC3 and analyze the interaction between this gene set and HDAC3 in LAML as well as its expression (Figure S1-A and Table 1). Next, we use STRING to draw a visual network diagram of the gene set expression (Figure S1-B). The results show that HDAC3 and myocyte enhancer factor 2D (MEF2D) have a strong coacting relationship (*p* < 0.05).

### 3.2. Enrichment Analysis of HDAC3 Functional Networks in LAML

As shown in the volcano map (Figure S2-A), dark green dots represent genes that are negatively associated with HDAC3 and dark red dots represent genes that are positively associated with HDAC3. The positive and negative correlations between 50 significant gene sets and HDAC3 were shown in the heat map (Figure S2-B, C). This result indicates that HDAC3 plays an important role in transcription. HDAC3 expression showed a strong positive correlation with SLC25A5 (positive rank #1, Pearson correlation = 0.67, *p* = 2.46*E* − 24), NDUFA2 (Pearson correlation = 0.67, *p* = 4.30*E* − 24), COX4I1 (Pearson correlation = 0.66, *p* = 8.30*E* − 23), and EIF3K (Pearson correlation = 0.65, *p* = 7.46*E* − 22); in addition, these genes have different effects on the production of energy and precursor metabolic molecules, mitochondrial material transport, and protein translation, which indirectly reflects that HDAC3 also plays a regulatory role in these cellular biological processes (Table 2). WebGestalt was used to conduct the GO annotations and to identify the main biological process (metabolic process and biological regulation), cellular component (nucleus), and molecular function (protein binding) related to HDAC3 biology (Figures 4(a)–4(c)). Kyoto Encyclopedia of Genes and Genomes (KEGG) pathway analysis showed that HDAC3 was directly involved in the thyroid hormone signaling pathway, while MEF2D, which had a synergistic relationship with it, was directly involved in the cGMP-PKG pathway (Figures 4(d) and 4(e)).

### 3.3. HDAC3-Targeting Drugs

We used the GDSC website to find a drug that targets HDAC3—entinostat. This study evaluated the growth inhibition effect of entinostat on acute myeloid leukemia cell lines in vitro. Entinostat had good inhibitory effects on all 17 cell lines, with the best inhibitory effect on LAML cell line MOLM-13 and the worst inhibitory effect on NOMO-1, with area under the curve (AUC) values greater than 0.5 (Table 3). A comparison of the half-maximal inhibitory concentration (IC50) values of the drug against different tumor cells showed that entinostat exhibited broad-spectrum antitumor activity in most tumors (Figure 5). Since the target gene of entinostat includes HDAC3, it has a certain antitumor effect on tumors with high HDAC3 expression, such as LAML.

## 4. Discussion

Acute myeloid leukemia has become the third leading cancer threat to human health today [24–26]. It is characterized by the rapid proliferation of abnormal cells in the bone marrow, which affects the production of normal hematopoietic cells.

Our study found that HDAC3 expression is increased in some types of acute myeloid leukemia, which may be associated with a shorter survival time. We hypothesized that the elevated expression of HDAC3 and the dysfunction of HDAC3 in acute myeloid leukemia might be caused by the structural changes of genes. HDAC3 has a variety of important physiological functions, and its alteration can cause the abnormality of a variety of signaling pathways. In acute myeloid leukemia, the gene network adjacent to HDAC3 also changes to a different degree. The related functional network is involved in cellular respiration, energy derivation by oxidation of organic compounds, tricarboxylic acid cycle, etc. Therefore, HDAC3 is closely related to gene transcription, protein translation, material transport, and cell growth.

Studies have shown that more than one-third of all LAML cases are caused by mutations in FLT3 kinase in myeloid cells [27–29]. Mutations in FLT3, an irritant growth factor receptor, can affect normal hematopoietic cell function, leading to abnormal cell proliferation and activation. We used UALCAN data analysis to show that HDAC3 expression was increased in patients with FLT3 mutations, and Novotny-Diermayr et al. have shown that certain HDAC inhibitors inhibit the expression of FLT 3 in LAML cells and thus treat LAML [30]. We suggest that HDAC3 may be a potential LAML therapeutic target to indirectly reduce FLT3 expression by reducing HDAC3 expression in LAML patients, which is worthy of further clinical validation.

Resistance to chemotherapeutic agents, which upregulate HDAC3 expression in LAML cells, is a major cause of poor prognosis in LAML cells [31]. Our study found that HDAC3 is directly involved in the thyroid hormone signaling pathway, which is one of the essential signaling pathways for regulating growth, development, and energy metabolism of the body. Thyroid hormones play an important role in the growth and differentiation of leukemia cells [32]. Thyroid hormone action is mediated by a variety of thyroid hormone receptor subtypes, and uncoated thyroid hormone receptors inhibit transcription by synthesizing a HDAC3-based inhibitor complex [33, 34]. Therefore, in acute myeloid leukemia, HDAC3 upregulation may inhibit the differentiation of leukemia cells through the thyroid hormone signaling pathway, leading to poor prognosis of the disease.

In this study, we also observed a synergistic gene MEF2D with HDAC3 and KEGG pathway analysis showed that MEF2D was directly involved in the cGMP-PKG signaling pathway. The cGMP-PKG signaling pathway can downregulate the expression of transcriptase, and its abnormal expression is closely related to the expression of the tumor suppressor gene p53 protein and the cell cycle inhibitor p21 [35, 36]. Mountains in p53 in acute myeloid leukemia are directly associated with overall survival (OS) in LAML patients [37, 38]. Therefore, we speculated that p53 and p21 may be important targets of MEF2D and MEF2D has a synergistic relationship with HDAC3 and HDAC3 can indirectly regulate the expression levels of p53 and p21 in LAML patients. Future research could further test this hypothesis.

HDAC can remove acetyl groups from the amino terminus of lysine residues on histones, while histone acetyltransferases (HATS) promote the addition of lysine residues, leading to structural changes in local chromatin [8, 39–41], which is an important step in regulating protein entry into DNA [7]. Studies have shown that HDAC and HATS enzymes are involved in the regulation of transcription factors, transcription modulators, and DNA repair proteins [42]. Abnormal expression of HDAC or abnormal recruitment of oncogenic proteins is present in many types of tumors, especially leukemia, and all of these conditions may contribute to the development of leukemia [43]. In response to the abnormal expression of HDAC3 in acute myeloid leukemia, we identified a HDAC3 inhibitor called entinostat. Recent studies have shown that entinostat induces apoptosis in LAML cells by restoring the expression of leukemia-associated transcription factors and proapoptotic proteins [36]. It has been confirmed that HDAC3 negatively regulates a transcription program associated with cytotoxic effects on CD8+ T cells and the selective HDAC3 inhibitor RGFP966 can strongly enhance the cytotoxic function of CD8+ T cells [44]. Our study also found that HDAC3 can block the mature differentiation of leukemia cells through certain signaling pathways. But the treatment of acute myeloid leukemia (AML) is not satisfactory. Histone deacetylase inhibitors (HDACi) have antileukemic cell activity both in vitro and in vivo [31, 45]. Clinical data suggest further testing of these epigenetic agents and the identification of mechanisms and markers of their efficacy. In conclusion, HDAC3 inhibits apoptosis induction and disrupts the expression of tumor-related proteins, thus playing a role of targeted therapy [46]. HDAC3 inhibitors, as a possible therapeutic drug, will provide some reference value for the treatment of acute myeloid leukemia to explore its specific mechanism of action.

One exciting therapeutic application of epigenetic therapy is in combination with adoptive cell therapy (ACT), including chimeric antigen receptor T cell (CAR T cell) therapy [47, 48]. HDAC inhibitors have been shown to promote the efficacy of ACT, which increases T cell recruitment at the tumor site. Preclinical trials of ACT showed that adoptive transfer of TSCM cells and TCM cell populations were significantly more effective than conventional use of Teff and T cell persistence was enhanced. Since T cell preservation in a tSCM-like state enhances the therapeutic effect, these processes are controlled by epigenetics, so it is possible to use epigenetic therapy to promote T cell “dryness” during lymphocyte expansion prior to reflux [49]. TET2 is a potential immunomodulatory target because unintentional insertion of CAR cDNA into the TET2 gene leads to the preservation of CAR T cells in TCM cell phenotypes and the clonal amplification of these cells. Therefore, it is suggested that potentially transient TET2 knockout or CAR T cell reexpression of TET2 may be advantageous in antigen-activated tumor sites. These studies highlight the potential for improvements in epigenetic therapies [50].

## 5. Conclusions

Although most of the drugs currently used to treat acute myeloid leukemia produces adverse outcomes, the treatment of LAML is dominated by chemotherapy. Therefore, finding new treatment methods is beneficial to improve the survival rate of patients and improve the quality of life after recovery. In recent years, increasing studies have tended to target therapy and research on LAML mutation genes has made continuous progress. According to the genetic mutation of LAML patients, tumor cells can be targeted to kill, while the function of normal cells is not affected. Among them, the abnormal expression of the target gene HDAC3 may affect the occurrence and development of LAML from different aspects, such as the cellular and molecular mechanism of action and its involvement in the regulation of signal transduction pathways. In the future, further exploration of the target gene HDAC3 and the development of corresponding targeted drugs will bring new hope for the treatment of LAML patients.

## Figures and Tables

**Figure 1:** HDAC3 expression in LAML (Oncomine). The copy number of HDAC3 mRNA and DNA in acute myeloid leukemia was significantly higher than that in normal tissues. Based on the Oncomine database analysis, the difference multiples and *p* values for cancer compared with normal tissue is shown. (a–d) Box plots show the mRNA expression levels of HDAC3 in Andersson leukemia, Valk leukemia, Stegmaier leukemia, and Haferlach leukemia data sets, respectively; (b) *p* value is less than 0.5. (e) Box plot shows the copy number of HDAC3 in TCGA.

**Figure 2:** HDAC3 transcription in subgroups of patients with LAML, stratified based on gender, age, and other criteria (UALCAN). (a) Box plot shows the relative expression of HDAC3 in patients with different subtypes of LAML M0, M1, M2, M3, M4, M5, M6, and M7. (b) Box plot shows the relative expression of HDAC3 in men and women. (c) Box plot shows the relative expression of HDAC3 in LAML patients aged 21–40, 41–60, 61–80, or 80–100 years. (d) Box plot shows relative expression of HDAC3 in Caucasian, African-American, or Asian LAML patients. (e) Box plot shows the relative expression of HDAC3 in the presence and absence of FLT3 mutation.

**Figure 3:** Effects of HDAC3 on survival time in LAML patients and its expression in pan-carcinomas. (a) Relationship between HDAC3 and survival time of LAML patients. The death rate of LAML patients increased over time, *p* < 0.05. (b) Comparison of HDAC3 expression in various types of cancer. Blue shows the expression level of HDAC3 in normal precancelled tissues, and red shows the expression level of HDAC3 in corresponding cancerous tissues.

**Figure 4:** Functional enrichment analysis of the HDAC3 gene (WebGestalt). (a–c) The main molecular functions, biological processes, and cell components related to the biology of HDAC3 were identified by the GO database. (d) KEGG annotation of the thyroid hormone signaling pathway. (e) KEGG annotation of the cGMP-PKG pathway.

**Figure 5:** Pharmacomics of HDAC3 (GDSC). (a) Semi-inhibitory concentrations of entinostat in different LAML cell lines. (b) AUC of the drug entinostat in different LAML cell lines. Based on GDSC database analysis, 17 LAML cell lines were used in the acute myeloid leukemia assay for this drug. The maximum and minimum IC50 or AUC values of the cell lines are shown. (c) IC50 values of entinostat in different types of tumor cells.

**Table 1:** Interaction between HDAC3-related gene sets and HDAC3.

Gene A	Gene B	Log2 odds ratio	*p* value	Tendency
HDAC3	SLC35A4	>3	<0.001	Cooccurrence
HDAC3	PFDN1	>3	<0.001	Cooccurrence
HDAC3	PSMB10	>3	<0.001	Cooccurrence
HDAC3	MEF2D	>3	0.012	Cooccurrence
HDAC3	TRIM6	>3	0.024	Cooccurrence
HDAC3	NUCB2	>3	0.024	Cooccurrence
HDAC3	DBNL	>3	0.058	Cooccurrence
HDAC3	PSMD4	>3	0.058	Cooccurrence
HDAC3	ZNF486	<-3	0.920	Mutual exclusivity
HDAC3	NUP93	<-3	0.942	Mutual exclusivity
HDAC3	SDHA	<-3	0.953	Mutual exclusivity
HDAC3	FH	<-3	0.953	Mutual exclusivity
HDAC3	ZNF826P	<-3	0.953	Mutual exclusivity
HDAC3	ZNF93	<-3	0.953	Mutual exclusivity
HDAC3	OXA1L	<-3	0.965	Mutual exclusivity
HDAC3	ATP5F1B	<-3	0.976	Mutual exclusivity
HDAC3	SLC25A5	<-3	0.988	Mutual exclusivity
HDAC3	ATP5F1A	<-3	0.988	Mutual exclusivity
HDAC3	ZNF665	<-3	0.988	Mutual exclusivity
HDAC3	NDUFS2	>3	1.000	Cooccurrence
HDAC3	SSBP3	>3	1.000	Cooccurrence
HDAC3	CST7	>3	1.000	Cooccurrence
HDAC3	EMID1	>3	1.000	Cooccurrence
HDAC3	ZNF566	>3	1.000	Cooccurrence

**Table 2:** The involvement of HDAC3-related gene sets in cellular biological processes.

Gene set	Description	Size	Enrichment ratio	*p* value	User ID
GO:0045333	Cellular respiration	175	17.82545	6.63*E* − 05	NDUFS2; SDHA; FH; OXA1L
GO:0009060	Aerobic respiration	80	29.24489	1.41*E* − 04	SDHA; FH; OXA1L
GO:0005746	Mitochondrial respiratory chain	89	26.28754	1.93*E* − 04	NDUFS2; SDHA; OXA1L
GO:0070469	Respiratory chain	99	23.63223	2.65*E* − 04	NDUFS2; SDHA; OXA1L
GO:0015980	Energy derivation by oxidation of organic compounds	261	11.95193	3.08*E* − 04	NDUFS2; SDHA; FH; OXA1L
GO:0006099	Tricarboxylic acid cycle	33	47.26446	8.09*E* − 04	SDHA; FH
GO:0006101	Citrate metabolic process	34	45.87433	8.59*E* − 04	SDHA; FH
GO:0072350	Tricarboxylic acid metabolic process	38	41.04545	0.001073	SDHA; FH
GO:0015932	Nucleobase-containing compound transmembrane transporter activity	39	39.99301	0.00113	SLC25A5; SLC35A4
GO:1901505	Carbohydrate derivative transmembrane transporter activity	41	38.04213	0.001249	SLC25A5; SLC35A4

**Table 3:** The antiproliferation effect of HDAC3 inhibitor entinostat on different cell lines.

Cell line	TCGA classification	Tissue	Tissue subtype	IC50 (*μ*M)	AUC
NOMO-1	LAML	Blood	Acute_myeloid_leukaemia	8.864915	0.893741
ME-1	LAML	Blood	Acute_myeloid_leukaemia	6.100197	0.865691
OCI-AML2	LAML	Blood	Acute_myeloid_leukaemia	4.978733	0.87515
ML-2	LAM	Blood	Acute_myeloid_leukaemia	3.566309	0.825786
KMOE-2	LAML	Blood	Acute_myeloid_leukaemia	3.472474	0.8081
KG-1	LAML	Blood	Acute_myeloid_leukaemia	3.175775	0.799341
HEL	LAML	Blood	Acute_myeloid_leukaemia	2.635879	0.78934
CESS	LAML	Blood	Acute_myeloid_leukaemia	2.313575	0.752965
OCI-AML5	LAML	Blood	Acute_myeloid_leukaemia	2.225316	0.771939
GDM-1	LAML	Blood	Acute_myeloid_leukaemia	2.080637	0.728326
HL-60	LAML	Blood	Acute_myeloid_leukaemia	1.916459	0.739312
CTV-1	LAML	Blood	Acute_myeloid_leukaemia	1.856703	0.748986
OCI-M1	LAML	Blood	Acute_myeloid_leukaemia	1.512284	0.713888
OCI-AML3	LAML	Blood	Acute_myeloid_leukaemia	0.703545	0.606781
KY821	LAML	Blood	Leukemia	0.649042	0.600801
KASUMI-1	LAML	Blood	Acute_myeloid_leukaemia	0.57003	0.581201
MOLM-13	LAML	Blood	Acute_myeloid_leukaemia	0.458012	0.552496

## Data Availability

All data generated or analyzed during this study are included in this published article.

## Abbreviations

AUC: Area under the curve
AKT: Protein kinase B
BP: Biological process
CC: Cellular component
CNV: Copy number variation
DNA: Deoxyribonucleic acid
FLT3: FMS-like tyrosine kinase 3
GDSC: Genomics of Drug Sensitivity in Cancer
GEO: Gene Expression Omnibus
GO: Gene Ontology
HATS: Histone acetyltransferases
HDAC: Histone deacetylase
HDAC3: Histone deacetylase 3
HDACi: Histone deacetylase inhibitors
IC50: Half maximal inhibitory concentration
KEGG: Kyoto Encyclopedia of Genes and Genomes
LAML: Acute myeloid leukemia
MEF2D: Myocyte enhancer factor 2D
MF: Molecular function
mRNA: Messenger RNA
MYC: Myeloma oncogene
TCGA: The Cancer Genome Atlas
WT1: Wilms tumor 1.

## Supplementary Materials

Supplementary 1 Figure S1: visual summary of HDAC3 gene alterations and coexpression networks of interacting gene sets in LAML (cBioPortal). (A) oncoPrint outlines the effect of HDAC3 genomic alterations on a single LAML sample from TCGA. The different types of mutations are shown in different colors. (B) Gene network view of HDAC3 in LAML. We selected 14 genes with a positive association with HDAC3 (selected with a threshold greater than 0.52) and 10 genes with a negative association (selected with a threshold of −0.34). The gene interactions were analyzed from the STRING database. The black line represents the coexpression relationship between the two genes. The blue line indicates the association in curated databases between two genes. The green line indicates the neighborhood in the genome. Yellow lines indicate two genes comentioned in PubMed abstracts. The purple line represents experimental/biochemical data between the two genes. (C) Heat map of transcriptional expression of 25 genes in acute myeloid leukemia.

Supplementary 2 Figure S2: LAML associated with HDAC3 differentially expressed genes set correlation studies (LinkedOmics). (A) The correlation between HDAC3 and LAML gene differential expression was analyzed by the Pearson correlation test. A negative value means a negative correlation, while a positive value means a positive correlation. A larger absolute value means a greater correlation. (B–C) heat maps showed the top 50 positively and negatively associated HDAC3 gene sets in LAML, respectively.
